# Construction of a Public Health-Oriented Sports Training Big Data Analysis Platform

**DOI:** 10.1155/2022/1788797

**Published:** 2022-08-23

**Authors:** Shangqi Nie

**Affiliations:** School of Physical Education, HuangHuai University, Zhumadian, Henan 463000, China

## Abstract

Sports health has become a goal pursued by most people, both young and old, which is mainly due to the improvement of people's living standards and the improvement of economic level. Different groups have great differences in the way of physical exercise for public health. The idea of pursuing physical exercise is better but most ignore the factors that affect exercise. Not only will this have a certain negative impact on body function but it also defeats the purpose of physical exercise. Reasonable physical exercise is more urgently needed. However, for public health physical exercise, reasonable methods are also difficult to obtain. This is mainly due to the large differences in the number of groups and hurdles faced by public health. This study designs a public health-oriented sports training platform based on big data technology. It mainly uses the hollow convolutional neural network (A-CNN) and the GRU method to extract the relationship between physical training and physical function, weather factors, and exercise intensity. The research results show that the A-CNN and GRU methods can better map the relationship between sports training parameters and the three characteristics that affect sports health. This kind of sports training platform based on big data technology can better guide young people or the elderly to carry out reasonable physical exercise. A-CNN and GRU techniques have relatively high accuracy in predicting the three characteristics of physical exercise. The smallest error is only 1.43%, and the largest error is also 2.56%.

## 1. Introduction

With the continuous improvement of living standards, people's pursuit of life has undergone great changes. In the past, people only pursued basic necessities of life, but now people are constantly pursuing good health and a happy life. Physical exercise has become an essential part of people's lives [1, 2]. People's pursuit of physical health is mainly divided into two reasons. The first is the continuous pursuit of physical health. The second is the improvement of living conditions, which leads to the improvement of the level of food. This further leads to obesity, which is the reason for the constant pursuit of physical fitness. Different groups have different reasons for pursuing physical fitness [3, 4]. For young people, the main reason for their pursuit of physical fitness is for a more perfect body. Sometimes, it's also a hobby. For the elderly, the main reason for their pursuit of physical fitness is to improve their physical function and health. Physical fitness can not only improve physical function, it can also keeps people in a happy mood. It can be said that sports health has become a pursuit of the people. With the continuous development of public sports health, there are also many types of physical exercise places and activities that further promote the development of public sports health. Improving public sports health has also become a task of the government. Different groups have different ways of exercising [5, 6]. Young people tend to focus on ball games or gym sports, which are quantitative exercise methods. They use high-tech technology to supervise their exercise process, which is also a scientific way of exercise. However, the elderly often use public sports equipment or walking as a form of physical and healthy exercise, and they rarely participate in high-intensity physical exercise. It also showcases a diverse sporting pattern. No matter what kind of sports group or what kind of healthy sports mode one chooses, scientific exercise methods are also more important [7, 8]. Scientific exercise methods not only protect your body, but also make sports and healthy exercise achieve the best exercise effect. High-intensity physical exercise not necessarily has a better effect. There is a strong relationship between public health physical exercise and physical function, weather, intensity, and other factors. A reasonable public health campaign method is more important, which requires more successful cases for reference. For physical exercise, most people do not understand the rationality of physical and healthy exercise. They rarely pay attention to the relationship between their physical function and the weather and exercise intensity. Reasonable public physical exercise methods and intensity are more critical for young people and the elderly. The parameters of this successful public sports training method need to be provided by professional sports personnel. Therefore, it is important to establish the relationship between the relevant data of sports training and physical function, exercise intensity, and weather factors.

It can be seen from the above description that most of the groups participate in more physical exercise in today's era in order to pursue more perfect physical health. However, they rarely notice the relationship between physical function and exercise intensity and weather factors. They perform public sports and health exercises according to their own hobbies and needs. They also pay little attention to the way they exercise. This will not only have a certain negative impact on the body, but also make it difficult to achieve the purpose of public sports and health campaigns. Proper exercise requires the advice of professional sports trainers or the reference of more successful case parameters to carry out related public physical exercises. The elderly often find it difficult to obtain the help of more professional sports personnel. Most of the elderly only exercise through simple ball games or walking. Most young people only perform physical exercise according to their own interests [9, 10]. Most people pay little attention to the relationship between the effect of public physical exercise and physical function, weather factors, and exercise intensity. Physical exercise has more influencing factors. However, physical function, weather factors, and exercise intensity are the three most influential characteristics, which are also relatively direct influencing factors. Therefore, the parameters of a common physical fitness exercise pattern are important for different sports groups. The collection of these motion parameters is difficult for most groups of motion, which requires a general motion parameter or platform as a relevant reference. Big data technology has developed rapidly and can be used to discover the relationship between exercise parameters and physical function, weather factors, and exercise intensity. These three factors are relatively objective factors. If these factors are not quantified, it is difficult to find the relationship between these factors and motion parameters. The amount of data related to the physical function and exercise intensity of physical exercise is huge, and the relationship between these three and the parameters of physical exercise is also complicated, which is very difficult for manual methods to compute. Thus, big data technology is exactly used to evaluate the advantage of this aspect.

Big data technology has developed rapidly in recent years. It is a research hotspot in today's era, and also solves many problems in many fields [11, 12]. Big data technology can handle huge amounts of data. For research objects and research tasks with a large amount of data, manual processing will consume a lot of time and human capital. With the development of computer technology, the characteristics of research objects can be converted into forms of data [13, 14], and big data technology can bring great advantages to production and life, and it can also realize the automation of technology. At the same time, big data technology has developed many mature algorithms, which have high stability and practicability in many fields. This is good news, as researchers only need to make minor adjustments as needed. Therefore, big data technology can also be applied to data in public health sports training. Currently, the most utilized algorithms are convolutional neural networks (CNN) and long short-term memory (LSTM) neural networks and reinforcement learning. The main role of CNN is to deal with spatial features between data and it can also map the relationship between different features. LSTM mainly deals with some temporal feature relationships. In life or production, temporal and spatial features are two common features. CNN and LSTM methods also contain more variant algorithms depending on the application environment. A-CNN is a variant of the CNN technology. GRU is a variant of the LSTM method. Both A-CNN and GRU techniques can reduce the amount of parameters in physical exercise-related operations. This also requires less computing resources.

This study mainly uses the atrous convolutional neural network (A-CNN) and the GRU neural network in big data technology to deal with the relationships between the huge amounts of data in public health sports training. The A-CNN method can map the relationship between physical exercise parameters and physical function, exercise intensity, and weather, while GRU can better extract the time features included between exercise intensity and weather. This study presents and analyzes the whole research from 5 different directions.  Section 1 illustrates the research significance of sports training in public health settings and the research background of big data technology. The research status of the factors related to physical training is studied in Section 2. The system scheme and related algorithms of the big data platform for public health sports training are studied in Section 3.  Section 4 presents the feasibility of the A-CNN and GRU methods in sports training research.  Section 5 summarizes the application value of the A-CNN and GRU methods in a public health-oriented sports training platform.

## 2. Related Work

In today's era, public physical exercise has also become a relatively popular recreational activity and has also produced more related industries and researches on physical exercise corresponding to public health. However, there is a lack of a public health-oriented physical training platform to guide the physical exercise of most groups. Of course, many researchers have studied the factors associated with physical activity. Pu [15] believed that sports videos will help the analysis of sports process by analyzing the process in the form of video playback. This improves the quality of movement and proposes a new motion video analysis method to address the shortcomings of the existing motion video analysis methods. It also describes the detailed video analysis process, and also conducts a comprehensive test on the motion video system; the research results show that this new motion video analysis method can capture the image of the video and also the effective information of the video. This accuracy has also been greatly improved. This method has certain practical value for guiding sports. Wang et al. [16] mainly improved the decision-making ability of sports players according to the training effect of sports. Their model devises a method of using association for sports running decision support system. It establishes a sports spatial motion model to analyze the distribution relationship of association rules. The methods of data mining and cloud computing are also used to fully mine the effect of sports operation. When mining sports training feature data, it adopts a method of fuzzy information fusion and data reorganization. It tests these methods in real training data mode. The research results show that this method has strong mining and decision-making abilities for sports training. Wang and Huang [17] believed that rehabilitation training of sports is a mode of restoring physical training, which can also restore related functions of the body. This is a beneficial training mode for the physique of the physical trainer and the prevention of diseases. It mainly uses intelligent algorithms to realize the health monitoring system of sports recovery training. They designed an intelligent sports health monitoring system, and it has also tested this health monitoring system in the actual recovery training. The research results show that this intelligent recovery training system can have good accuracy, with an accuracy of 92.6%. This intelligent recovery training health monitoring helps protect the health of trainers. Wang et al. [18] mainly focus on some sports training and physical exercises during summer camps or exchange visits, which is also a common sports exchange and public sports health problem. They developed and designed a sports training program, and these sports-related activities are mainly related to overseas markets. The model determines the factors that affect this sports mode according to the current situation of the relevant literature, which provides a reference for the development of sports training programs. Fu [19] has collected sports training data using wireless sensor technology, and also carried out in-depth research on the collected data. The researcher designed an athlete data collection system according to the needs of sports trainers, which includes data collection terminals and wireless sensors and other technologies. The model will realize real-time collection and analysis of athlete training data. The research results show that this system collects first data and improves the training performance by 16%. This system can meet the needs of athletes' training data collection and storage, which will also be of great value to athletes' data analysis. Wang [20] has realized the importance of training assistance systems for sports training, and hence used an improved machine learning algorithm to study training-aided decision-making systems for physical exercise. This applies maximum entropy and adversarial neural network techniques to sports training samples. The introduction of this algorithm can solve the problem of uneven edge distribution of sports training data. It also applies this decision-making system to actual sports training. The research results also verify the importance and reliability of this decision-making system for sports training. Current research rarely uses the A-CNN and GRU methods to study the relationship between physical exercise parameters and physical function and exercise intensity. Once this relationship is established, it can better guide different groups to carry out efficient physical exercise.

## 3. Application Scheme of the A-CNN and GRU Methods in Sports Training Big Data Platform

### 3.1. The Significance of Big Data Technology for the Prediction of Physical Exercise Characteristics

Through the above introduction, it can be found that the physical functions of physical exercise, exercise intensity, and weather factors are the key factors that affect physical health. However, the characteristics of these three factors are difficult to find by artificial means. There are also different relationships between the physical health of different groups and these three factors. This brings fewer references to physical exercise for different groups. Excessive exercise intensity and exercise in bad weather are both detrimental to health [21]. However, artificial methods are unable to establish the relationship between physical function, weather factors, and exercise intensity and physical fitness. There is a complex relationship between these factors and physical health. This requires the application of big data technology. The big data technologies selected in this study are A-CNN and GRU. They can comprehensively consider the problem of feature extraction and calculation time. A-CNN can save more parameter computation than CNN technology, and it can also extract features efficiently. The biggest advantage of big data technology is the processing of complex data, which is also a major disadvantage of manual methods. In general, big data technology can not only help people find the relationship between physical health and physical function, exercise intensity, and weather factors, it can also predict unknown factors, which can be very good to guide different groups to perform physical exercise.

### 3.2. Design Principles of A-CNN and GRU in Sports Training Big Data Platform

The ultimate goal of this research is to design a sports training big data platform, which is mainly aimed at public health sports. This is also to solve the problem of the lack of relevant parameters and technical guidance in the public health model. Considering the huge amount of parameters of the physical exercise big data platform, it adopts the variant neural network A-CNN of CNN. At the same time, it also takes into account the strong relationship between weather characteristics and exercise intensity characteristics and time, and it uses the GRU method. Both of these methods can reduce the amount of parameter computation to a certain extent.  Figure 1 shows the design flow of the sports training big data platform using the A-CNN method as well as the GRU method. The characteristics here mainly include physical function, exercise intensity, and weather factors. Although there is a certain correlation between physical training and other characteristics, the influence of these three factors is relatively large and intuitive. The collection and processing of the dataset is the most critical step, which will affect the training accuracy and convergence. This flowchart is not shown. The data of these three features once collected will be used as the input data of A-CNN. The data will go through the convolutional layers, pooling layers, and activation functions of A-CNN. When the relevant features are learned, the data will then go through the GRU in a sequence, where the temporal features of the three features are extracted. A-CNN will establish the relationship between sports parameters and the three influencing factors. The output data of A-CNN is the input data of GRU again as a sequence. Finally, the GRU outputs the physical exercise health index through the output layer. There is a feedback propagation mechanism in the calculation of output and loss of physical exercise. The output and loss are continuously affected at each iteration step.

CNN has been applied in many fields as it can reduce the amount of parameter computation compared to fully connected neural networks. However, if the number of layers of CNN reaches a certain level, it will still have more parameters. This results in wasted computing resources and time. With the continuous progress of CNN methods, atrous convolutional A-CNN technology has shown better performance in extracting features. It has less parameter computation compared to traditional CNN methods. This is advantageous for large datasets.  Figure 2 shows the workflow of A-CNN in the sports training big data platform, which is similar to that of CNN. The difference is that there will be fewer parameters in the convolution layer during the convolution operation.

### 3.3. The Principle and Introduction of the A-CNN and GRU Equation

The computational complexity of the LSTM method is large, and it will consume more time and computing resources. This is bad for deeper network layers. In order to reduce the number of parameters of the LSTM, researchers have discovered the GRU algorithm, which is also good at dealing with time problems.  Figure 3 shows the application process of the GRU method in the sports training big data platform. Compared with the LSTM, the gate structure is changed from 4 to 2. Although the number of gate structures is reduced, it can still effectively process historical information as well as current information. It can also efficiently output historical information related to current state information. It can be seen from Figure 3 that the structure of GRU is relatively simple compared to the LSTM. However, the performance of GRU does not degrade on large datasets. There is a certain similarity in structure between the GRU and LSTM methods. The difference is that the number of gate structures is different, and there is also a certain gate structure calculation in the hidden layer of GRU. However, the reset gate of GRU and the forget gate of the LSTM have a similar role as the input gate.

It can be clearly seen from Figure 3 that GRU also has two gate structures, which are update gate and reset gate, respectively. Compared with the LSTM, it has two less gate structures. The hidden layer unit of GRU also introduces a gate structure, which can assist in the memory and selection of information.

Equations (1) and (2) show how the reset gate of the GRU is calculated. The reset gate will replace the LSTM's forget gate and input gate. It will also re-select and input the input information and historical information according to the size of the weight.

(1) $$\begin{array}{c} g_{r}=\sigma \left(W_{r}\left[h_{t-1},x_{t}\right]+b_{r}\right), \end{array}$$

(2) $$\begin{array}{c} \tilde{h_{t}}=\tan\;h\left(W_{h}\left[g_{r}h_{t-1},x_{t}\right]+b_{h}\right). \end{array}$$

Equations (3) and (4) show the calculation criteria for the update gate of the GRU. It is similar in function to the output gate and update gate of the LSTM. It will continuously update the information that needs to be output according to the size of the weight.

(3) $$\begin{array}{c} g_{\text{z}}=\sigma \left(W_{z}\left[h_{t-1},x_{t}\right]+b_{z}\right), \end{array}$$

(4) $$\begin{array}{c} h_{t}=\left(1-g_{z}\right)h_{t-1}+g_{z}\tilde{h_{t}}. \end{array}$$

Equations (5) and (6) show the method of derivation calculation for weights and biases. For A-CNN and GRU, this derivation method exists in each layer of their structure. Although the operations of the two methods are different, Equations (5) and (6) are general calculation guidelines.

(5) $$\begin{array}{c} \Delta \omega_{ji}=-\eta \frac{\partial E}{\partial \omega_{ji}}, \end{array}$$

(6) $$\begin{array}{c} \Delta u_{ij}=-\eta \frac{\partial E\;\partial }{\partial u_{ij}}. \end{array}$$

For A-CNN, the output size of features is somewhat different from CNN. This is also related to the convolution operation form of the hidden factor. Equation (7) shows how the output feature size of A-CNN features is calculated.

(7) $$\begin{array}{c} S_{\text{out}}=\left\lfloor \frac{S_{\text{in}}+2\text{pading}-S_{\text{kenal}}}{\text{step}}\right\rfloor +1. \end{array}$$

In A-CNN, if there is a deconvolutional neural network, it is not impossible to obtain the original size; it needs to go through a certain convolution operation to obtain the original feature size. Equation (8) shows how the original feature size is calculated by deconvolution. Equation (9) shows a calculation criterion for the receptive field.

(8) $$\begin{array}{c} S_{\text{in}}=\left(S_{\text{out}}-1\right)\times \text{step}+S_{\text{kenal}}-2\text{pading,} \end{array}$$

(9) $$\begin{array}{c} V_{i}=V_{i-1}+S_{\text{kenal}-i}\times \prod_{i=1}^{i-1}{\text{step}}_{i-1}. \end{array}$$

Equation (10) shows the activation function used in this study, which is typically placed in the last layer of the neural network. It will non-linearize the extracted features. Otherwise, all data will be output in a linearized manner.

(10) al=ReLUzl=ReLUWlal−1+bl.

The loss function is a function that exists in every neural network structure, and it is also a driving force for gradient descent methods. Most loss functions use the mean square error function. Equation (11) shows the mean square error function used in this study, which will calculate the error between the predicted and actual values of the physical training parameters. Gradient descent will use this error to find the smallest gradient direction.

(11) $$\begin{array}{c} L=\text{MSE}\left(q^{\text{real}},q^{\text{pre}}\right)=\frac{1}{nm}\sum_{k=1}^{N}\sum_{j=1}^{M}{\left(q_{kj}{}^{real}-q_{kj}{}^{pre}\right)}^{2}. \end{array}$$

## 4. Result Analysis and Discussion

This study uses the A-CNN and GRU methods in the field of big data to design a sports training monitoring intelligent system for national health. It mainly solves the problem of lack of relevant data reference in the field of public health sports. The A-CNN method is used to extract relevant features of physical training, and it is also used to map the relationship between physical training parameters and training-related factors. This study mainly selected three characteristics: physical training, weather factors, and exercise intensity. The GRU method mainly extracts the temporal features of these three factors. This is also because weather factors and bodily functions are constantly changing over time. At the same time, the forming the dataset is also an important process. In this study, relevant sports training data and physical exercise parameters in Beijing were selected as the training and test sets. In order to ensure the accuracy of the test set, the test set of this study was also derived from the actual data. Not only does Beijing have a high population density, but the movement patterns here are diverse, and datasets with more features can also be collected.

In this paper, the A-CNN and GRU methods have been selected as methods for evaluating the sports training big data platform. The advantages of these two methods vary. A-CNN can extract features between physical function, exercise intensity, and weather factors. GRU mainly extracts the time relationship of these three. In order to verify the validity of the GRU method and verify the weather factors and the correlation between physical function and time, this study first used a single A-CNN method for training and testing.  Figure 4 shows the error distribution of the three effects of physical training. In Figure 4, V1 represents the physical performance feature of physical exercise. V2 represents the exercise intensity feature related to physical exercise. V3 represents the characteristics of weather influencing factors. On the whole, the prediction errors obtained using a single A-CNN method can also meet the needs of the sports training big data platform, and the three prediction errors are all distributed within 3.5%. However, the prediction errors of these three influencing factors all exceed 2%, which is unfavorable for the accuracy and stability of the sports training big data platform. This shows that the features of the three factors are not fully extracted. This limits the application of the sports training big data platform in real life. From this point of view, A-CNN cannot fully meet the needs of the sports training big data platform for accuracy and reliability.

Since a single A-CNN method cannot meet the needs of a sports training big data platform, it is necessary to consider the temporal correlation of physical exercise. After all, physical exercise is a long-term process, which is closely related to time. This study further predicts and analyzes these three factors using a hybrid A-CNN and GRU method.  Figure 5 shows the prediction error of the three factors of the sports training big data platform using the A-CNN and GRU methods. The red line indicates that the prediction errors of the three characteristics of physical exercise are within the 2% interval. This will divide the prediction error by a 2% bound. This more clearly sees the effect of A-CNN and GRU. From Figure 5, it can be seen intuitively that the prediction errors of the three factors have been greatly reduced. This not only shows the importance of the GRU method to the sports training big data platform, but also further shows that the three factors of sports training have strong temporal correlation. When using the sports training big data platform, it is necessary to fully consider the time correlation. Prediction errors for both physical function and exercise intensity were reduced to less than 2%. The prediction error of physical function is 1.78%, while the prediction error of exercise intensity is only 1.43%. This is extremely accurate and reliable for the sports training big data platform. The forecast errors of weather factors remained at a high level, which may be related to the lack of data in the dataset.

The above analysis analyzes the relative accuracy of the sports training big data platform through the average prediction error. It selects 30 different sets of data to introduce the prediction distribution of the three factors of physical training.  Figure 6 shows a scatterplot of prediction errors for physical performance features in the sports training big data platform. Overall, most of the scatterplot data are distributed within 2% of the data for the 30 groups of physical performance characteristics. Only one set of data has an error of more than 2%. However, the magnitude of excess is also relatively small. This fully shows that the A-CNN and GRU methods have extremely high accuracy in predicting the special physical function of the sports training big data platform, which is beneficial for practical applications. There were also two groups with prediction errors of less than 1% for physical performance characteristics. If the A-CNN and GRU methods are applied in actual training, they can accurately predict the relationship between physical function factors and physical exercise parameters.

Similarly, this study still selected 30 sets of data to analyze the prediction of exercise intensity using the A-CNN and GRU methods.  Figure 7 shows the distribution of the predicted value and the actual value of the exercise intensity feature of the sports training big data platform. Exercise intensity is an important parameter for physical exercise, and the prediction accuracy of this parameter will determine the time and type of physical exercise. This is also a physical exercise feature that can be easily grasped. On the whole, the eigenvalues of exercise intensity predicted by the A-CNN and GRU methods are consistent with the actual values regardless of the magnitude of the value or the change trend of exercise intensity. Although there are obvious fluctuations in the eigenvalues of exercise intensity, there are many peaks and troughs between two adjacent eigenvalues of exercise intensity. However, A-CNN and GRU still show better performance, which predicts the fluctuation of motion intensity better. This is better reliable for the application of the actual sports training big data platform.

The influence of weather factors on physical exercise is a relatively objective factor. However, it also has a greater impact on the effect of physical exercise. The weather factor has great variability, and its prediction in the sports training big data platform is also relatively large. This study chooses the form of box plot to show the effect of A-CNN and GRU in predicting weather factors.  Figure 8 shows the box plot of the predicted and actual values of weather features in the sports training big data platform. A box plot can not only show the magnitude of the values, it can also show the distribution of two sets of values. On the whole, the predicted box distribution of weather factors is relatively consistent with the actual box distribution. The data value of the weather factor obtained by the A-CNN-GRU methods is relatively large, but the error between the two is relatively small. From the mean point of view, the distribution of the two is also smaller. Overall, the A-CNN-GRU methods can more accurately predict the weather characteristics in the sports training big data platform.

## 5. Conclusions

People's pursuit of life is constantly improving, and physical exercise is one of the more important manifestations. Physical exercise can not only improve physical health, it can also improve the happiness index of life. Both young and old have their own patterns of physical activity, mostly for their own hobbies and health. However, they paid little attention to the level of physical fitness that physical activity achieves. This is also because there are fewer parameters for them to compare and guide. This limits the purpose of physical exercise in public health. Physical exercise must have a certain scientific basis. It needs to carry out reasonable physical exercise according to factors such as physical function and weather. It is not that the greater the intensity of physical exercise, the better. Different groups have different levels of physical activity. This requires physical exercise parameters in a public health model for their reference.

This research uses the A-CNN and GRU methods in big data technology to design a physical exercise big data platform. It mainly uses the A-CNN and GRU methods to predict factors that are more relevant to physical exercise. This study mainly selected physical function, exercise intensity, and weather factors as the research objectives. For a single A-CNN method, although it can accurately predict the three characteristics of the physical exercise big data platform, the prediction errors of these three characteristics are also within a reasonable range. However, the prediction errors of factors such as physical function and exercise intensity are relatively high, which lacks certain reliability for the practical application of the physical exercise big data platform. For the hybrid A-CNN and GRU model, the prediction errors of physical function, running intensity, and weather factors are significantly reduced. The error of physical function and exercise intensity is less than 2%. The largest prediction error is only 2.56%, which is also related to the variability of weather factors. In general, the application of the A-CNN and GRU methods in the physical exercise big data platform is feasible, and it also has relatively high stability.

## Figures and Tables

**Figure 1:** Design principles of A-CNN and GRU in the sports training big data platform.

**Figure 2:** The working principle of the A-CNN algorithm.

**Figure 3:** The working principle of the GRU method.

**Figure 4:** Prediction errors for the three features in the sports training platform utilizing a single A-CNN approach.

**Figure 5:** Prediction errors of the three features in the sports training platform using the A-CNN and GRU methods.

**Figure 6:** Distribution of scatter plots of the prediction errors for physical function.

**Figure 7:** Distribution curve of the predicted value and the actual value of the exercise intensity feature.

**Figure 8:** Prediction of weather characteristics of the sports training big data platform and box plot distribution of actual values.

## Data Availability

^*∗*^The dataset can be accessed upon request.
